The article "Research on Sino Japanese Comparative Literature from the Perspective of Sustainable Ecological Environment" was retracted in 2023. Reasons: unreliable results or conclusions; concerns about the data; concerns about the results or conclusions; concerns about the peer review.

# Research on Sino Japanese Comparative Literature from the Perspective of Sustainable Ecological Environment

**DOI:** 10.1155/2022/5396135

**Published:** 2022-06-21

**Authors:** Quan Fang

**Affiliations:** School of Foreign Languages and Literature, Shandong University, Jinan 250100, Shandong, China

## Abstract

**Objective:**

This study promotes the comparison and research of Chinese literature and Japanese literature from the perspective of the ecological environment of sustainable development.

**Methods:**

This study analyzes and compares the differences in the literary cultures of different countries. After the analysis, it is found that the literary culture has never been solid and conservative. We should look at the national literary culture and national differences from the perspective of development.

**Results:**

The results show that in the research of Chinese and Japanese comparative literature from the perspective of a sustainable ecological environment, it is found that through the comparison and analysis of concept differences, thinking differences, behavior differences, and language differences in Chinese and Japanese comparative literature, it can be seen that Chinese literature has a more far-reaching impact on national quality education than Japanese literature, which is more progressiveness and has a reference value.

**Conclusion:**

The analysis and research of Chinese and Japanese comparative literature cannot be underestimated in promoting the development and progress of the country, and it can provide a good foundation for promoting the establishment of a bridge of friendly exchange between Chinese and Japanese nationalities so as to shorten the distance between each other.

## 1. Introduction

The sustainable development of the ecological environment is closely related to the development of the social economy. The ecological environment provides essential resources for human survival and development. The Chinese nation has always respected and loved nature. The 5000 year old Chinese civilization is pregnant with a rich ecological culture. The prosperity of ecology leads to the prosperity of civilization, and the decline of ecology leads to the decline of civilization. Civilization is the historical accumulation of culture, and culture is the external manifestation of civilization. The development process from agricultural civilization to industrial civilization to ecological civilization is also a process of continuous deconstruction and reconstruction of the ecological culture paradigm [1]. Ecological culture is the spiritual achievement of the harmonious development between man and nature, the spiritual link of maintaining the relationship between man and nature, and the spiritual force of building ecological civilization. China has entered a new era, comprehensively promoting the construction of economic, political, cultural, social, and ecological civilization. Its foundation is the construction of ecological civilization, and what guides the construction of ecological civilization is ecological culture. The development of cultural industry is an important part of national construction. With the rapid development of the social economy, all countries have begun to pay attention to the construction of cultural industry [2]. The ecological culture of different civilization backgrounds has its own typical characteristics in essence, theory and method. A profound grasp of the transformation law of ecological culture is the internal requirement for accurately grasping the essence of the construction of ecological civilization.

The article "Research on Sino Japanese Comparative Literature from the Perspective of Sustainable Ecological Environment" was retracted in 2023. Reasons: unreliable results or conclusions; concerns about the data; concerns about the results or conclusions; concerns about the peer review.

If a country's cultural development wants long-term and progress, it is necessary to correctly grasp the relationship between national literature and world literature. The construction of national literature is inseparable from the theory and method of comparative literature [3]. The literature of each nation should not become a closed and independent individual but should be understood and analyzed from the perspective of comparison and influence. Since modern times, there has been a relatively close exchange between Chinese literature and foreign literature. It is found that literary works of different countries have their own characteristics. It is not clear which is better or worse on the macro level. It can only be said that each has its own merits. Therefore, the literary works of any country have reading value and should be analyzed accordingly [4]. Literary works are not only the crystallization of language, but also record the history and social changes of a country. Literature is the product of worldwide circulation. Comparative literature studies a country's literary phenomena and related cultural phenomena from the perspective of borderlessness. Comparative literature puts the literature of various countries into this overall structure for understanding and comparison, and reveals and grasps the laws and relations of literature. The gradual deepening of reform and opening up and the all-round development of the economy have built a good environment for the development of Chinese culture, which has led to the rapid development of China's comparative literature research. Chinese and Japanese comparative literature has become a hot field of comparative literature research [5]. China and Japan are neighbors separated by a strip of water. With the migration of history and the precipitation of time, the two countries have both similarities in culture and different cultural characteristics [6]. In ancient times, from the dispatch of Sui envoys, the monks entering the Song Dynasty, Confucianism in the Tang Dynasty, and the custom of drinking tea in the Song and Yuan Dynasties were introduced into Japan. In terms of material and spiritual aspects, China was comprehensively affecting Japan and improving its social development and progress. In modern times, Japan's development was faster than that of China. When China lagged behind the world, it also got the influence of Japan and indirectly the advanced civilization of the west through Japan. From the communication of Chinese language and characters to clothing and means of transportation, China and Japan influenced and contrasted each other in their existing customs and cultures.

The article "Research on Sino Japanese Comparative Literature from the Perspective of Sustainable Ecological Environment" was retracted in 2023. Reasons: unreliable results or conclusions; concerns about the data; concerns about the results or conclusions; concerns about the peer review.

## 2. An Analysis of the Current Situation of Comparative Literature between China and Japan

The exchange history of Chinese and Japanese literature is bounded by the Meiji Restoration, and the comparative literature research between China and Japan is carried out from the two fields of Chinese and Japanese ancient literature and Chinese and Japanese modern literature. The important achievement of Chinese and Japanese comparative literature is the comparative study of Chinese and Japanese ancient literature. Since Japan entered the Meiji Restoration, Western culture has been continuously introduced into Japan, which became a new thing and a turning point in the trend of Japanese literature, leading to the rise of Japanese modern literature [7]. In the early 1980s, a group of scholars such as Jiang Xijin, Lin Huanping, and Sun Xizhen began to study the relationship between Chinese new literature and Japanese modern literature, which is also the backbone of Chinese and Japanese modern comparative literature research. The comparative study of Chinese and Japanese modern literature has taken a completely different path from the comparative study of Chinese and Japanese ancient literature. Because of the enlightenment of Japanese modern literature to Chinese modern literature, the foothold of Chinese modern literature is Chinese modern literature. Although the characters in Japanese literature and culture evolved from Chinese characters, great changes have taken place in the writing and content expression after a long time of development and change. For foreign literature and culture, we should always maintain a modest attitude, learn and think, “take the essence and discard the dross.” Since the 1990s, there have been a number of influential works on comparative literature. For example, Wang Xiangyuan's comparative theory of Chinese and Japanese modern literature has found some new problems in Chinese and Japanese modern literature from a new perspective. Zhang Fugui and Jin Conglin's comparative study of Chinese and Japanese modern literary relations clearly and comprehensively combs the history of Chinese and Japanese modern literary relations and exchanges in the order of historical occurrence, and Hu Lingyuan's resonance and development of civilization—A Study of Sino Japanese cultural relations, The book discusses the significance of Japanese literature to modern Chinese literature and reflects on Chinese and Japanese culture. Cross-cultural interpretation pursues equal exchanges and mutual learning between different cultures, so it plays a positive role in the external communication of Chinese culture [8]. Ting correctly understands the interaction between different literature, which is of great significance for absorption, sublation, and innovation after influence. Only in this way can we correctly understand the national characteristics of their respective literature and have prominent significance in the study of Chinese and Japanese comparative literature [9].

The article "Research on Sino Japanese Comparative Literature from the Perspective of Sustainable Ecological Environment" was retracted in 2023. Reasons: unreliable results or conclusions; concerns about the data; concerns about the results or conclusions; concerns about the peer review.

## 3. Analysis of the Differences in Various Aspects of Chinese and Japanese Comparative Literature

### 3.1. Conceptual Differences between Chinese and Japanese Comparative Literature

Culture is borderless and excellent. No matter which country it is from, it can be used for reference and recognized by all countries in the world. However, culture is different, and different countries and regions have distinctive characteristics in all aspects [10]. Conceptual differences are reflected in the process of subtle influence and the influence of the surrounding environment. They are formed through observation, learning, and personal experience. They are generated from a specific culture and have their own views, judgment, and attitude towards things. Therefore, concept is not only the criterion of people's daily life and activities but also a yardstick to judge their words and deeds. The main reason for the conceptual difference between Chinese and Japanese comparative literature is that China has always believed in Confucianism since ancient times, with “benevolence” as the core of the thought. After Confucianism spread to Japan, it chose “ceremony” as the core thought. This is the initial reason for the formation of the concept difference of comparative literature between China and Japan, but Japan's literature and culture lack the thickness of inheritance. China's literature and culture have experienced thousands of years of precipitation and accumulation. The thought has long been deeply rooted, and the ideological depth has long reached an unreachable height. Through the comparison of the differences in the concept of comparative literature between China and Japan in terms of national cohesion, family honor, and personal values, this paper analyzes, discusses, and studies the two different literary and cultural directions of Chinese literature and Japanese literature as shown in Table 1.

The article "Research on Sino Japanese Comparative Literature from the Perspective of Sustainable Ecological Environment" was retracted in 2023. Reasons: unreliable results or conclusions; concerns about the data; concerns about the results or conclusions; concerns about the peer review.

In Table 1, through the analysis of the conceptual differences between Chinese and Japanese comparative literature under the two different literary and cultural directions in the above table, it can be seen that in terms of national cohesion and personal values, Chinese literature has a higher influence on the people than Japanese literature. In terms of family honor, Japanese literature has a deeper impact on the people than Chinese literature.

In order to better reflect the comparison results of the conceptual differences between Chinese and Japanese comparative literature under the analysis of two different literary and cultural directions, the data comparison results in Table 1 are visualized, and Figure 1 is obtained.

Figure 1 shows the comparison results of the conceptual differences between Chinese and Japanese comparative literature under the analysis of two different literary and cultural directions. Chinese literature has far more influence on the people in terms of national cohesion and personal values than Japanese literature. Japanese literature has a higher influence on the people in terms of family honor than Chinese literature. The influence of Chinese literature and culture on their nationals is broader than that of Japanese literature and culture and has better ideological guidance for their nationals. It shows that in different aspects, two different literary cultures have their own strengths and weaknesses.

### 3.2. Thinking Differences between Chinese and Japanese Comparative Literature

The thinking difference is reflected in the problem and implementation, as well as in the logical ability. The ability is improved by forming independent systematic thinking, which gradually opens the thinking gap in these processes. Therefore, thinking is the reflection of people's brain on objective reality. It is a unique spiritual activity of people, which is produced from a large number of social practices. The main reasons for the formation of the thinking difference between Chinese and Japanese comparative literature is because of the country's region, the country's productivity, and the country's unique cultural thought. China has a vast region, rich and diverse resources, and a unique national culture; however, Japan's territory is narrow, the types of resources are scarce and limited, and most of its national culture is a mixture of learning from and accepting the cultural ideas of other foreign countries. Therefore, China's literature and culture has the style of a big country, while Japan's culture is relatively chaotic and complex. Under the influence of this literary thought, Japanese people's thinking mode is more conservative and old-fashioned. By comparing the thinking differences of Chinese and Japanese comparative literature in terms of national self-discipline, interpersonal relationship and communication mode, and analyzing, discussing, and studying the two different literary and cultural directions of Chinese literature and Japanese literature, Table 2 is obtained.

The article "Research on Sino Japanese Comparative Literature from the Perspective of Sustainable Ecological Environment" was retracted in 2023. Reasons: unreliable results or conclusions; concerns about the data; concerns about the results or conclusions; concerns about the peer review.

In Table 2, through the analysis of the thinking differences between Chinese and Japanese comparative literature under the two different literary and cultural directions in the above table, it can be seen that in the three aspects of national self-discipline, interpersonal relationships, and interpersonal communication mode, Chinese literature has a higher influence on the people than Japanese literature and a deeper influence than Japanese literature.

In order to more intuitively reflect the comparison results of thinking differences between Chinese and Japanese comparative literature under the analysis of two different literary and cultural directions, the data comparison results in Table 2 are visualized, and Figure 2 is obtained.

Figure 2 shows the comparison results of the conceptual differences between Chinese and Japanese comparative literature under the analysis of two different literary and cultural directions. The influence and influence of Chinese literature on the people in the three aspects of national self-discipline, interpersonal relationships, and interpersonal communication mode are far greater than that of Japanese literature. It shows that Chinese literature and culture are more suitable as the thinking guidance of the people and are more conducive to the development of national conditions.

### 3.3. Behavioral Differences between Chinese and Japanese Comparative Literature

The fundamental reason for the formation of the difference between Chinese and Japanese comparative literature is Confucianism, but the reason for the formation of the behavior difference between Chinese and Japanese comparative literature is also composed of other factors, such as geographical environment, national geographical location, and so on, which lead to great differences in people's behavior and activities. Behavioral differences are reflected in the innate physiological quality and social environment. Through later education and social practice activities, they show different behaviors and activities dominated by ideas. The basic reason for the formation of the difference between Chinese and Japanese comparative literature is Confucianism, but the reason for the formation of the behavioral difference between Chinese and Japanese comparative literature is also composed of other factors, such as the geographical environment and location of the country, which lead to great differences in people's behavior and activities. Through the comparison of thinking differences between Chinese and Japanese comparative literature in terms of integrity consciousness, time concept consciousness, and work attitude consciousness, and through the analysis, discussion, and research of the two different literary and cultural directions of Chinese literature and Japanese literature, Table 3 is obtained.

The article "Research on Sino Japanese Comparative Literature from the Perspective of Sustainable Ecological Environment" was retracted in 2023. Reasons: unreliable results or conclusions; concerns about the data; concerns about the results or conclusions; concerns about the peer review.

In Table 3, through the analysis of the thinking differences between Chinese and Japanese comparative literature under the two different literary and cultural directions in the above table, it can be seen that Japanese literature has a higher influence on people than Chinese literature in terms of time concept consciousness and work attitude consciousness. In the sense of honesty, Chinese literature has a deeper influence on people than Japanese literature.

In order to more intuitively see the behavioral difference comparison results of Chinese and Japanese comparative literature under the analysis of two different literary and cultural directions, the data comparison results in Table 3 are visualized, and Figure 3 is obtained.

Figure 3 shows the comparison results of the conceptual differences between Chinese and Japanese comparative literature under the analysis of two different literary and cultural directions. Japanese literature has a better influence on the people in terms of time awareness and work attitude awareness than Chinese literature. Chinese literature has a deeper influence on the people in terms of integrity consciousness than Japanese literature. It shows that different literary cultures have different emphases on the influence of people's behavior. Each country has its own literary culture and behavior mode, which cannot be generalized.

### 3.4. Language Differences between Chinese and Japanese Comparative Literature

The differences in the way of thinking and culture are reflected in the differences in the way of thinking and life. The main reasons for the language differences between Chinese and Japanese comparative literature is the differences in the use of vocabulary and the specific ways of language expression. Through the comparison of thinking differences between Chinese and Japanese comparative literature in terms of vocabulary differences, language differences, and expression methods, this paper analyzes, discusses, and studies the two different literary and cultural directions of Chinese literature and Japanese literature, and obtains Table 4.

The article "Research on Sino Japanese Comparative Literature from the Perspective of Sustainable Ecological Environment" was retracted in 2023. Reasons: unreliable results or conclusions; concerns about the data; concerns about the results or conclusions; concerns about the peer review.

In Table 4, through the analysis of the thinking differences of Chinese and Japanese comparative literature under the two different literary and cultural directions in the above table, it can be seen that in terms of vocabulary differences and language differences, Chinese literature has a higher influence on the people than Japanese literature. In terms of differences in expression, Japanese literature has a deeper impact on the people than Chinese literature.

In order to more intuitively reflect the behavior difference comparison results of Chinese and Japanese Comparative Literature under the analysis of two different literary and cultural directions, the data comparison results in Table 4 are visualized, and Figure 4 is obtained.

Figure 4 shows the comparison results of the conceptual differences between Chinese and Japanese comparative literature under the analysis of two different literary and cultural directions. Chinese literature has a better influence on the people than Japanese literature in terms of vocabulary differences and language differences. The influence of Japanese literature on the people in terms of differences in expression is deeper than that of Chinese literature. It shows that although the characters in Japanese literature and culture evolved from Chinese characters, great changes have taken place in the writing and content expression after a long time of development and change. For foreign literature and culture, we should always maintain a modest attitude, learn and think, “take the essence and discard the dross.”

## 4. Discussion

Both China and Japan have long literary and cultural traditions. With the background of opening to the outside world and the development of global integration, cultural exchanges between countries are becoming more and more frequent. With the joint efforts of China and Japan, the literary relations between the two countries have developed rapidly. Although the two countries have various differences in the mode of cultural inheritance, it is undeniable that the national cultures of China and Japan affect and permeate each other. Wang Z recalled that in the 20th century, the study of Chinese and Japanese comparative literature has experienced a long period of exploration and rapid development, and has made good achievements. Looking forward to the 21st century, the study of Chinese and Japanese comparative literature has been advancing on the road of vigorous development [11]. From the birth of comparative literature to the formation of the Chinese School reflects the change of research direction and the continuous expansion of the research vision of comparative literature. Although Chinese comparative literature started relatively late, it is playing an increasingly important role on the stage of world comparative literature [12]. No matter how the world changes, the cultural foundation of Chinese literature and Japanese literature cannot be changed. Their national aesthetics and values inherit the tradition in progress and revise and develop it in inheritance. Chinese comparative literature develops slowly under the background of globalization. In its development process, it not only maintains unique Chinese characteristics but also draws lessons from the experience of comparative literature development in other countries, so that Chinese comparative literature in the new period can adapt to the development of the new era.

The article "Research on Sino Japanese Comparative Literature from the Perspective of Sustainable Ecological Environment" was retracted in 2023. Reasons: unreliable results or conclusions; concerns about the data; concerns about the results or conclusions; concerns about the peer review.

## 5. Summary

At present, all countries are facing the trend of sustainable ecological development and global integration. The integrated sustainable development will no longer be embodied in one aspect, but in all-round common development and progress in many aspects, and the cornerstone and focus of national development is the country's unique culture and literacy. This study makes a detailed analysis and discussion on the differences in all aspects of Chinese and Japanese comparative literature from the perspective of sustainable ecological environment. By comparing the differences in concept, thinking, behavior and language of Chinese and Japanese comparative literature, and using statistical methods to express the research of Chinese and Japanese comparative literature more intuitively, it can be seen that the differences of Chinese and Japanese comparative literature have different effects on their nationals. The enthusiasm of the people of the two countries for literature and learning has increased greatly. They learn from the strengths of the comparative literature of the two countries and learn from the weaknesses of their own comparative literature, which provides a more favorable scheme for sustainable ecological development and speeds up the pace and process of sustainable development of global integration.

## Figures and Tables

**Figure 1:** Visualization of conceptual differences between Chinese and Japanese comparative literature.

**Figure 2:** Visualization of thinking differences in Japanese comparative literature.

**Figure 3:** Visualization of behavioral differences between Chinese and Japanese comparative literature.

The article "Research on Sino Japanese Comparative Literature from the Perspective of Sustainable Ecological Environment" was retracted in 2023. Reasons: unreliable results or conclusions; concerns about the data; concerns about the results or conclusions; concerns about the peer review.

**Figure 4:** Visualization of language differences between Chinese and Japanese comparative literature.

**Table 1:** Conceptual differences between Chinese and Japanese comparative literature.

Group	National cohesion (%)	Family honor (%)	Personal values (%)
Chinese literature	95.40	79.60	87.30
Japanese literature	89.60	92.80	76.90

**Table 2:** Data of thinking differences in Japanese comparative literature.

Group	National self-discipline (%)	Interpersonal relationship (%)	Interpersonal style (%)
Chinese literature	94.20	86.40	91.30
Japanese literature	87.60	78.20	88.70

**Table 3:** Data table of behavioral differences between Chinese and Japanese comparative literature.

Group	Honesty consciousness (%)	Time concept consciousness (%)	Work attitude awareness (%)
Chinese literature	93.90	78.20	86.40
Japanese literature	86.30	86.90	92.80

**Table 4:** Data of language differences between Chinese and Japanese comparative literature.

Group	Lexical differences (%)	Language differences (%)	Expression differences (%)
Chinese literature	96.20	94.60	89.10
Japanese literature	83.20	84.90	91.80

## Data Availability

The data underlying the results presented in the study are available within the manuscript.
